The article "Implication of Salivary Biochemical Parameters for Diagnosis and Prognosis of Type 2 Diabetes Mellitus" was published in 2022. Journal: Int J Anal Chem.

# Implication of Salivary Biochemical Parameters for Diagnosis and Prognosis of Type 2 Diabetes Mellitus

**DOI:** 10.1155/2022/1781613

**Published:** 2022-08-10

**Authors:** Sneha Shrestha, Sushant Pokhrel, Anjali Poudel, Shristi Bhandari BC, Mudita Shakya, Alaska Timilsina, Manisha Sapkota, Bashu Dev Pardhe

**Affiliations:** Department of Laboratory Medicine, Manmohan Memorial Institute of Health Sciences, Kathmandu, Nepal

## Abstract

**Background:**

Clinical laboratory diagnosis and prognosis for diabetes mellitus is performed using blood as a major specimen; however, saliva may represent as an alternative noninvasive specimen of choice. This study aims to evaluate salivary biochemical parameters in diabetic and healthy individuals to substantiate saliva's role in the diagnosis and prognosis of type 2 diabetes mellitus (T2DM).

**Methods:**

This case-control study included 150 T2DM patients and 150 apparently healthy individuals. Socio-demographic data and anthropometric measurements were recorded using a standard questionnaire. Correlation between salivary and blood levels for each parameter was determined using Pearson correlation. Linear regression was performed to estimate the blood levels of the parameters from their salivary levels. Receiver operating characteristics (ROC) analysis was done to determine the diagnostic ability of salivary glucose and establish a sensitivity, specificity, and cut-off value.

**Results:**

Salivary glucose, TC, LDL-C, urea, and creatinine were significantly higher in people with diabetes than in the control population (*p* < 0.05). A significant positive correlation was found between salivary and blood parameters including glucose, TC, TG, LDL-C, urea, and creatinine except for HDL-C in both case and control groups. The linear relationship for each parameter, except glucose in case population and HDL-C in case, control, and the total population was observed between blood and saliva. ROC analysis gave a cut-off value of 1.9 mg/dl for salivary glucose with 71.4% sensitivity and 72.3% specificity.

**Conclusion:**

Salivary estimation significantly reflects the blood parameters in this study, indicating that saliva can be a noninvasive specimen for the diagnosis and prognosis of T2DM.

## 1. Introduction

Diabetes mellitus (DM) is a chronic, noncommunicable disease evolving at a startling pace around the world. Morbidity and mortality in diabetes are due to a steady rise in hyperglycemia and manifestation of associated complications such as cardiovascular disorder, nephropathy, retinopathy, neuropathy, and lower extremity amputations. Frequent screening, early-stage diagnosis, and resolute management of diabetes have become a major requirement to lower diabetes incidence globally [1, 2].

The article "Implication of Salivary Biochemical Parameters for Diagnosis and Prognosis of Type 2 Diabetes Mellitus" was published in 2022. Journal: Int J Anal Chem.

Standard diagnostic tests for diabetes as proposed by International Diabetes Federation (IDF) and World Health Organisation (WHO) include fasting or random or 2-hour glucose estimation following ingestion of 75-g glucose load assessment in plasma or HbA1c test [3]. Type 2 diabetes mellitus (T2DM) renders as an independent risk factor for dyslipidemia and kidney disease, which are responsible for morbidity and mortality among patients with diabetes due to the development of cardiovascular disease (CVD) and chronic kidney disease (CKD), respectively. Cardiovascular complications have the highest mortality rate among patients with diabetes. Management of healthy levels of lipids amongst them has shown to reduce both morbidity and mortality, increasing their quality of life. Hence, regular monitoring of lipid profile is a must over the course of the disease. Diabetic dyslipidemia characterized by abnormal serum lipid (elevated triglyceride, low-density lipoprotein cholesterol, and low high-density lipoprotein cholesterol) leads to CVD risk in patients with DM [4]. To prevent adverse cardiovascular outcomes in T2DM patients, assessment of CVD plays a pivotal role [5]. The proportion of CKD attributable to diabetes alone ranges from 12 to 55%. The incidence of CKD is up to 10 times higher in adults with diabetes than in those without [6]. Frequent analysis of renal function tests in patients with diabetes can decrease this incidence drastically.

Needle-associated anxiety and discomfort regarding frequent blood sampling are often detested and can prevent people from screening or monitoring their blood parameters [7]. Underlying conditions such as clotting factor deficiencies, compromised venous access, anemia, and the need for major vein preservation can also hinder the screening or monitoring process. Involvement of needle prick possess a potential risk for both patients and health care professionals towards blood-borne infections [8–10]. Avoidance of invasive procedures can reduce such infection risks.

Urine samples have been used in the prognosis of diabetes, but as the renal threshold for glucose is high, fasting conditions cannot be applied to urine as it accumulates in the bladder over time [1]. Here, saliva can be a simpler alternative whenever blood sampling is unsuitable or inaccessible. Noninvasiveness, ease of sampling, and cost-effectiveness can encourage frequent testing in patients for proper screening or management of the disease.

Saliva is a blood filtrate present as an extracellular body fluid in the oral cavity [11] The passage of blood constituents into saliva is due to transcellular, passive intracellular diffusion, active transport, or paracellular routes by extracellular ultrafiltration within the salivary glands or through the gingival sulcus [12, 13]. Various studies verify that the composition of saliva is affected by local or systematic changes. Systemic disease like DM notably alters the function of the salivary gland affecting the quality of saliva it produces [14]. Various studies indicate the usefulness of saliva for the estimation of glucose, lipid profile, urea, and creatinine in the diagnosis and prognosis of diabetes and its complications [8, 15–17]. A small molecule like glucose easily diffuses through a semi-permeable membrane into saliva. In DM, hyperglycemia leads to vascular defects resulting in an altered basement membrane of blood vessels. Even larger amounts of glucose and serum components can diffuse into saliva from the blood [9].

The article "Implication of Salivary Biochemical Parameters for Diagnosis and Prognosis of Type 2 Diabetes Mellitus" was published in 2022. Journal: Int J Anal Chem.

This study explores fasting unstimulated salivary biochemical parameters level and compares it with the blood level of biochemical parameters of significant complications related to T2DM such as glucose, lipid profile, urea, and creatinine. Other papers related to salivary parameters emphasize a single parameter or single profile [7, 8, 16]. Hence, these salivary parameters have not been assessed together in a single patient with DM or control population group, unlike in our study. Thus, this alternative noninvasive method will aid in early diagnosis as well as regular monitoring of diabetes to prevent complications by effective management of hyperglycemia.

## 2. Materials and Methods

### 2.1. Study Design and Population

This cross-sectional case-control study was conducted in Manmohan Memorial Teaching Hospital (MMTH) Kathmandu, Nepal for the period of six months (February 2020 to July 2020). A total of 150 already diagnosed T2DM patients attending the Department of Medicine and Endocrinology for the follow-up were conveniently selected for case population and 150 apparently healthy volunteers (hospital staff) were selected for the study as a control population.

#### 2.1.1. Inclusion and Exclusion Criteria

Patients clinically diagnosed with T2DM at least for 6 months were included as case population. Furthermore, age, sex, and BMI matched apparently healthy (free of DM, Metabolic diseases, and oral diseases) volunteers (hospital staff) were selected for the study as a control population. Population with any history of oral disease, salivary gland surgery, or any kind of oral/dental surgery and T2DM patients with insulin therapy were excluded from this study. Population under the long-term medication of any kind of disease, regular smokers, and alcoholics were also excluded. Patients with T1DM were not included in the study.

The article "Implication of Salivary Biochemical Parameters for Diagnosis and Prognosis of Type 2 Diabetes Mellitus" was published in 2022. Journal: Int J Anal Chem.

After informed and written consent, the population fulfilling the above criteria was recorded with demographic data such as age, gender, smoking history, alcohol consumption, undergoing medications, year of diagnosis of DM, diagnosis of patients with DM complication, frequency of blood parameters monitoring, and oral disease or oral surgical history.

### 2.2. Anthropometric and Blood Pressure Measurement

According to the guidelines of the WHO STEPS surveillance Manual, height, weight, waist circumference (WC), hip circumference (HC), and blood pressure were measured. Height and weight were measured without shoes, with patients standing erect on a portable height measuring board and digital weighing machine, respectively. A measuring tape was held above the light clothing of patients, at the maximum circumference over the buttocks for WC and around the maximum circumference of the buttocks for HC. Body mass index (BMI) was calculated (kg/m^2^) [18].

Blood pressure was measured using a sphygmomanometer from the left arm, placed on a desk with palm facing upward, with the antecubital fossa at level to the heart [18]. Hypertension was described as systolic blood pressure (SBP) above 140 mm of Hg or diastolic blood pressure (DBP) above 90 mm of Hg or a patient under treatment with hypertensive drugs [2].

### 2.3. Biochemical Analysis

Fasting (8 to 12 hours) unstimulated whole saliva and blood samples were collected for biochemical analysis. Saliva samples (3–5 ml) were collected in a sterile container by spitting method, after overnight fasting and rinsing the mouth with drinking water prior to collection. Patients were advised to sit in a restful, upright position with the head tilted slightly forward and mouth slightly open to pool saliva on the mouth floor. Talking, oral movements, and swallowing were refrained [15, 19]. Blood samples for glucose were collected in a sodium fluoride tube, and blood samples for lipid profile, urea, and creatinine were collected in a tube with a clot activator.

Saliva samples were centrifuged at 5000 rpm for 15 min, and the supernatant was separated and used for the test. Blood samples were centrifuged at 3000 rpm for 5 min to separate plasma/serum. Saliva supernatant and serum were stored at −20°C until further processing. Fasting saliva and blood samples were analyzed for glucose, total cholesterol (TC), triglyceride (TG), high-density lipoprotein cholesterol (HDL-C), urea, and creatinine as per the instructions provided by the reagent manufacturer (Human GmBh, Wiesbaden, Germany). All the parameters were analyzed using a HumaStar 300 (Human Diagnostics, auto-analyzer) in the Department of Biochemistry, MMTH.

The article "Implication of Salivary Biochemical Parameters for Diagnosis and Prognosis of Type 2 Diabetes Mellitus" was published in 2022. Journal: Int J Anal Chem.

### 2.4. Statistical Analysis

Data were analyzed using SPSS version 20.0 (IBM Corp., Armonk, NY, USA) and Microsoft Excel 2013. Salivary and blood parameters between patients with diabetes and healthy controls were compared using the independent samples *t*-test. Chi-square test was used to test for association between categorical variables. The Pearson correlation test was performed on both the study groups to observe linear relation between salivary and blood parameters and determine if a change in the salivary levels reflected blood level changes. Linear regression analysis was done to obtain an equation for estimation of the blood levels of the parameters from their salivary levels. A regression equation was obtained for each parameter as *y* (serum level) = *m* (regression coefficient) × *x* (salivary level) + *c* (constant). Regression coefficient gives an increase or decrease in serum parameter with a unit change in its salivary parameter. Receiver operating characteristics (ROC) analysis was performed to determine the diagnostic ability of glucose and to obtain a cut-off value for salivary glucose.

## 3. Results

This study comprised of 300 subjects, of which 150 were patients with diabetes, and 150 were apparently healthy individuals. The patients with DM population in our study included 71 males and 79 females, with a mean age of 55.86 ± 12.13 years, while 74 males and 76 females with a mean age of 52.4 ± 10.8 years were the control population. There was no significant difference in age, sex, waist circumference, hip circumference, and BMI among the patients with diabetes and controls. Systolic and diastolic blood pressure were found significantly higher in diabetes patients in comparison to the control group (Table 1).

The majority of diabetes patients had existing diabetic complications, and the average duration of diabetes diagnosis was 8.74 ± 8.11 yrs. Their clinical report assessment presented hypertension in 47% of patients with diabetes, followed by cardiovascular disease in 23%, renal dysfunction in 16%, retinopathy in 10%, and peripheral vascular disease in 4% of patients with diabetes as a complication (Table 1).

Needle-associated anxiety was present in 25% of the total population and 28% of the total patients with diabetes population. Irregularity of blood glucose monitoring was reported by 53% of the total population and 26% of the total patients with diabetes population (Table 2).

Glucose, TC, LDL-C, urea, and creatinine level were significantly higher in the saliva of the patients in DM population than of healthy individuals. Salivary TG and HDL-C showed no significant difference between the patients with DM and the control population. Furthermore, glucose, TG, urea, and creatinine showed significantly higher mean values in the serum of the patients with diabetes population compared to the control population (Table 3).

The article "Implication of Salivary Biochemical Parameters for Diagnosis and Prognosis of Type 2 Diabetes Mellitus" was published in 2022. Journal: Int J Anal Chem.

A significant positive correlation of salivary glucose, TC, TG, LDL-C, urea, and creatinine was established with their blood level in patients with DM as well as a control population. No significant correlation was found for HDL-C (Table 4).

Table 5showed a linear regression correlation between salivary parameters (glucose, TC, TG, LDL-C, urea, and creatinine) and blood parameters (glucose, TC, TG, LDL-C, urea, and creatinine) in case, control and total population. Linear regression analysis gave an equation for each parameter for all three case/control/total populations with a significant linear regression correlation, except for glucose in case population and for HDL-C in case and control population.

We tested the diagnostic potential of saliva compared to blood for diabetes by using ROC curve analysis (Figure 1). ROC analysis separated the whole population under study into those with and without the disease in question using blood glucose as a gold standard. The total area under the curve obtained for salivary glucose was 0.76 (standard error 0.05, *p*-value < 0.001, 95% CI 0.66–0.87). We established sensitivity and specificity for different values of salivary glucose, and a cut-off value of 1.9 mg/dl was determined as this gave the best trade-off with a sensitivity of 71.4% and specificity of 72.3%.

## 4. Discussion

Regular monitoring of blood parameters provides us with a prognosis of a disease and complications associated with it. In our previous report, we found that self-adherence to regular blood monitoring significantly reduces the HbA1c level in patients with diabetes [20]. Thus, keeping track of the extent of hyperglycemia and its complications in patients with diabetes is a crucial aspect. Regular monitoring of blood glucose, lipid profile, and renal function tests has been a key component of effective management and therapy of diabetes. Invasiveness of the blood sampling, associated with potential risks and anxiety, often hinders this monitoring process [1, 8, 10, 15]. Our study revealed that 26% of the diabetes population had irregularity of blood monitoring, and among them, 53.8% expressed needle-associated anxiety during their blood monitoring.

Lipid profile is one of the key prognostic markers for tracking the probable cardiovascular events among patients with diabetes. People with diabetes have compromised lipid metabolism and are said to have twice or thrice times higher risk of CVDs than those without diabetes [21]. In our study, salivary TC, LDL-C was significantly higher among patients with diabetes than in the control group. In contrast, there was no significant difference in salivary TG between patients with diabetes and the control group despite the significant difference in their serum levels. This may be due to partial action of lingual lipase acting upon salivary TG. In addition, a significant positive correlation between serum and salivary TC, TG, and LDL-C was observed in our study, which implies that their salivary level imitated their blood level. This finding opens up the possibility of the use of saliva for testing of these markers in the prognosis of CVDs in patients with diabetes. However, neither a significant decrease nor a positive correlation was found for HDL-C in saliva or serum between patients with diabetes and the control population in our study. Similar to our findings, lipid profile parameters in saliva are reported indiscriminately by other similar studies. Shivani et al. [22] found a significant rise in TC, TG, and LDL-C but not for HDL-C in both saliva and blood among patients with diabetes compared to controls, along with a significant positive correlation between their salivary and blood levels in both the groups. Whereas, Al-Rawi [16] presented significant elevation of TC, TG, LDL-C, and significant depletion of HDL-C in patients with diabetes in comparison to healthy controls alongside a significant positive correlation in the parameters in both study groups.

The article "Implication of Salivary Biochemical Parameters for Diagnosis and Prognosis of Type 2 Diabetes Mellitus" was published in 2022. Journal: Int J Anal Chem.

Besides cardiovascular complications, many patients with diabetes develop renal dysfunction in the course of diabetes, which is preventable. T2DM is among the leading cause of renal failure resulting from damage to podocytes and loss of filtration surface [23]. Urea and creatinine are primarily excreted by the kidneys, so any dysfunction in it can be indicated by elevated levels of urea and creatinine in body fluids. In our study, we explored the possibility of salivary urea and creatinine instead of their serum levels as a prognostic marker. Our result demonstrates a significant elevation of urea and creatinine levels in serum as well as in saliva in patients with diabetes compared to healthy individuals. A significant positive correlation between salivary-serum urea, and creatinine implies that their salivary level imitated their serum level. Pandya et al. [6] presented increased salivary urea and creatinine among patients with diabetes in comparison to healthy individuals in the study. Thereby, it is evident that salivary urea and creatinine can be used as an alternative to serum urea and creatinine.

Regular screening of glucose levels in the blood helps in the early diagnosis of T2DM and for estimation of the extent of hyperglycemia in patients with diabetes, which determines the course of the disease. Monitoring of hyperglycemia thus helps to prevent fatal complications that diabetes has to offer. The potential of salivary glucose for the diagnosis and prognosis of diabetes remains a debate. The present study finds a significantly elevated level of salivary glucose among the patients in DM group than in the healthy controls, and a significant positive correlation between salivary and blood glucose levels was established in both study groups. Many studies in concordance with our study reported a significant increase in salivary glucose in patients with diabetes compared to healthy individuals [1, 15, 17, 24]. However, some studies presented no increase in salivary glucose levels in patients with diabetes despite a rise in blood glucose levels [25, 26]. Carda et al. found a normal level of glucose among 76.4% of patients with diabetes with abnormal salivary glucose levels only for patients with DM population with poor metabolic control [26]. Various other studies have also found a significant positive correlation between salivary and blood glucose in the total study population [15, 17]. In contrast to our study, few other studies could not establish a correlation between saliva and blood glucose levels [25–27]. This may be due to the diversity of subject, study design, sample collection, and processing time as well as their storage conditions in these studies than in ours. LN Forbat et al. used stimulated saliva samples for their study in contrast to our unstimulated saliva sampling [25]. Similarly, Englander et al. also used stimulated saliva samples and a different testing method [27]. Studies have established that stimulation affects the production of saliva, altering its composition [14].

The article "Implication of Salivary Biochemical Parameters for Diagnosis and Prognosis of Type 2 Diabetes Mellitus" was published in 2022. Journal: Int J Anal Chem.

A significant positive correlation for parameters reinforces the likelihood of the use of saliva as a potential substitute for blood. The elevated level of parameters on saliva and positive correlation between their salivary and serum level might be due to diabetic microangiopathy. Microcirculation is associated with the delivery of nutrients into cells from the blood. Blood derivatives supposedly pass from blood in capillaries around salivary glands into saliva by transcellular, passive intracellular diffusion, and active transport, or by paracellular routes [12,13].

Persistence of hyperglycemia leads to increased nonenzymatic glycation of proteins and lipids and ultimately increased advanced glycation end products (AGEs). AGEs alter physical properties of protein in extracellular matrix by forming cross-links and by engaging receptors for AGEs (RAGE). AGE-bound RAGE increases endothelial permeability to macromolecules [28]. Prolonged hyperglycemia also induces sorbitol-myoinositol-mediated changes, redox potential alterations, and protein kinase C (PKC) activation. All of these biochemical changes manifest as structural changes that include capillary basement membrane (BM) thickening and vascular permeability [28, 29]. Increased permeability forms a leaky vasculature structure that leads to increased passage of blood components into saliva, simultaneously increasing the level of passed components in saliva with an increase in their blood level [15].

Linear regression analysis gave an equation for each parameter for all three case/control/total populations with a significant linear correlation except for HDL-C. No significant linear correlation was obtained for glucose in case population and for HDL-C in case and control populations. This may be due to our small study population size. Various other studies have found a linear relationship between serum and salivary glucose [15, 30]; and between serum and salivary urea [30]. To the best of our knowledge, no literature has reported linear regression analysis on lipid profile or creatinine.

Evaluation of salivary diagnostic tests in comparison to established standard diagnostic tests should be done to assess their practical usability. The accuracy of salivary diagnostic depends on its ability to separate the group being tested into diseased and healthy [31]. Thus, to establish salivary glucose as an alternative to gold standard blood analysis, ROC analysis was done, which gave the sensitivity and specificity of salivary measures. In our study, the cut-off value for salivary glucose was 1.9 mg/dl with a sensitivity of 71.4% and specificity of 72.3%. A study by Mrag M et al. found a cut-off value of 4.5 mg/dl (0.25 mmol/L) with 78% sensitivity and 80% specificity [30]. Khayamzdeh M et al. found a cut-off value of 1.05 mg/dl for unstimulated saliva in their study [32]. Another study by Smriti et al. established a cut-off point of 7.05 mg/dl, with a sensitivity of 99.1% and specificity of 93.7% [33]. So, there is an observation of a higher salivary glucose cut-off value for stimulated saliva compare to nonstimulated fasting saliva. Patients in our study were on regular medication, and fasting unstimulated saliva was analyzed, which might be the cause for our lower glucose value in saliva.

Our study limits in the sense that it was carried out with limited number of subjects. The time duration of onset of T2DM among patients was not considered during analysis, so the effect of progression of diabetes on salivary parameters could not be established. For saliva analysis, we used reagents and instruments designed to be used on serum samples. Furthermore, more sensitive methods for the detection of salivary glucose can be pivotal in the use of saliva for the diagnosis and prognosis of T2DM due to the low levels of parameters in saliva. W. Zhang et al. in their study, have introduced a noninvasive glucose monitoring method using a saliva nano-biosensor that can detect salivary glucose levels as low as 0.1 mg/dL and as high as 20 mg/dL [7]. This finding along with our results strengthens the foundation for the use of fasting unstimulated saliva in the diagnosis and prognosis of T2DM. The development of such sensitive technologies, preferably portable, can render saliva a desirable sample in a large number of screenings, diagnosis, and prognosis of T2DM.

The article "Implication of Salivary Biochemical Parameters for Diagnosis and Prognosis of Type 2 Diabetes Mellitus" was published in 2022. Journal: Int J Anal Chem.

## 5. Conclusion

The significant differences in salivary parameters between case and control and the significant positive correlation between salivary and blood glucose, total cholesterol, triglyceride, LDL-C, urea, and creatinine indicate that saliva reflects the blood values. Furthermore, we established the linear relationship between them in our study population except for glucose in case population and HDL-C. A cut-off value of 1.9 mg/dL was obtained with a sensitivity of 71.4% and specificity of 72.3% for salivary glucose. Based on our findings, we can suggest that unstimulated fasting salivary glucose, urea, creatinine, TC, TG, and LDL-C are worth exploring for their use as a screening, diagnostic and prognostic tool because of their potential. Saliva, being a noninvasive technique, can be easily used for frequent screening in patients to give us insight into the disease progression and in monitoring therapy and replace the use of blood in various point of care devices used for self-monitoring.

## Figures and Tables

**Figure 1:** Receiver operating curve for salivary glucose levels with total area under curve 0.76 with a sensitivity of 71.4% and specificity of 72.3%.

**Table 1:** Comparison of means of various demographic and anthropometric data between diabetic and healthy control.

Variables		Diabetic (*n* = 150)	Control (*n* = 150)	*p*
Age (years)		55.86 ± 12.13	52.4 ± 10.79	0.135
Gender	Male	71 (47.3%)	74 (49.3%)	0.841
	Female	79 (52.7%)	76 (50.7%)	
WC (cm)		90.48 ± 9.96	90.41 ± 12.19	0.975
HC (cm)		97.82 ± 9.68	96.18 ± 9.7	0.399
BMI (kg/m^2^)		26.02 ± 4.25	26.02 ± 3.76	0.995
SBP (mmHg)		121.3 ± 14.03	115.3 ± 9.5	**0.014**
DBP (mmHg)		78.8 ± 7.18	74.7 ± 6.73	**0.004**
HbA_1_ c (%)		7.16 ± 0.66	5.5 ± 0.27	**<0.001**
Duration of diabetes (years)		8.74 ± 8.11	—	—
Complication			—	—
Hypertension		72 (47%)		
CVD		36 (23%)		
Renal dysfunction		24 (16%)		
Retinopathy		15 (10%)		
PVD		6 (4%)		

WC, waist circumference; HC, hip circumference; BMI, body mass index; SBP, systolic blood pressure; DBP, diastolic blood pressure; CVD, cardiovascular disease; PVD, peripheral vascular disease; All the values expressed in mean ± SD; independent student's *t*-test used to analyze mean comparison; Chi-square test used to analyze the comparison between the categorical variable; Bold indicates the level of significance (*p* < 0.05).

The article "Implication of Salivary Biochemical Parameters for Diagnosis and Prognosis of Type 2 Diabetes Mellitus" was published in 2022. Journal: Int J Anal Chem.

**Table 2:** Needle associated anxiety and irregularity in blood monitoring in subjects.

	Total study population (*n* = 300)	Case (*n* = 150)		Control (*n* = 150)	
	No. (%)	No. (%)		No. (%)	
Needle associated anxiety	75 (25%)	42 (28%)		33 (22%)	

Irregularity in monitoring	159 (53%)	39 (26%)		120 (80%)	
		Needle associated anxiety			
		Yes	No	Yes	No
		21 (53.80%)	18 (46.20%)	30 (25%)	90 (75%)

Irregularity in monitoring refers to more than a month gap between blood testing.

**Table 3:** Mean comparison of salivary and blood biochemical parameters between patients with DM and control group.

Variable		Diabetic (*n* = 150)	Control (*n* = 150)	*p*
Glucose (mg/dl)	Salivary	2.74 ± 1.48	1.36 ± 0.55	**<0.001**
	Plasma	135 ± 41.72	89.2 ± 10.61	**<0.001**

TC (mg/dl)	Salivary	13.26 ± 7.03	8.58 ± 3.57	**<0.001**
	Serum	172 ± 52.22	161.15 ± 29.59	0.195

TG (mg/dl)	Salivary	10.95 ± 6.10	9.03 ± 3.76	0.062
	Serum	141.42 ± 68.22	108.9 ± 45.09	**0.006**

HDL-C mg/dl	Salivary	1.67 ± 0.79	1.34 ± 0.97	0.064
	Serum	44.25 ± 9.83	41.26 ± 9.33	0.122

LDL-C (mg/dl)	Salivary	9.39 ± 6.66	5.43 ± 3.62	**<0.001**
	Serum	99.47 ± 48.63	98.11 ± 26.51	0.863

Urea (mg/dl)	Salivary	37.23 ± 11.54	24.57 ± 7.34	**<0.001**
	Serum	32.61 ± 9.29	23.78 ± 5.42	**<0.001**

Creatinine (mg/dl)	Salivary	0.22 ± 0.13	0.13 ± 0.07	**<0.001**
	Serum	0.76 ± 0.27	0.63 ± 0.13	**0.004**

Tc, total cholesterol; TG, triglyceride; HDL-C, high-density lipoprotein cholesterol; LDL-C, low-density lipoprotein cholesterol; All the values expressed in mean ± SD; Independent student's t-test used to analyze mean comparison; Bold indicate the level of significance at *p* < 0.05.

**Table 4:** Correlation between salivary and blood biochemical parameters.

Variable		Groups	Pearson (r)	*p*-value
Salivary vs. Blood	Glucose	Diabetic	0.299^*∗*^	0.035
		Control	0.402^*∗∗*^	0.004
	TC	Diabetic	0.348^*∗*^	0.013
		Control	0.327^*∗*^	0.021
	TG	Diabetic	0.431^*∗∗*^	0.002
		Control	0.316^*∗*^	0.025
	HDL-C	Diabetic	0.091	0.531
		Control	0.244	0.087
	LDL-C	Diabetic	0.296^*∗*^	0.037
		Control	0.335^*∗*^	0.017
	Urea	Diabetic	0.625^*∗∗*^	<0.001
		Control	0.505^*∗∗*^	<0.001
	Creatinine	Diabetic	0.836^*∗∗*^	<0.001
		Control	0.602^*∗∗*^	<0.001

Tc, total cholesterol; TG, triglyceride; HDL-C, high-density lipoprotein cholesterol; LDL-C, low-density lipoprotein cholesterol. ‘R' denotes correlation coefficient; ^*∗*^indicate the level of significance at *p* < 0.05; ^*∗∗*^indicate the level of significance at *p* < 0.001.

The article "Implication of Salivary Biochemical Parameters for Diagnosis and Prognosis of Type 2 Diabetes Mellitus" was published in 2022. Journal: Int J Anal Chem.

**Table 5:** Table showing linear regression analysis of salivary and blood variables in total population.

Variable		Linear regression equation	*p*	*R* ^2^
Blood glucose	Total	*y* = 81.78 + 14.84 × (salivary glucose)	**<0.001**	0.262
	Case	*y* = 114.07 + 7.7 × (salivary glucose)	0.054	0.08
	Control	*y* = 78.8 + 7.69 × (salivary glucose)	**0.004**	0.16

Blood TC	Total	*y* = 139 + 2.52 × (salivary TC)	**<0.001**	0.133
	Case	*y* = 137.7 + 2.58 × (salivary TC)	**0.01**	0.12
	Control	*y* = 140 + 2.47 × (salivary TC)	**0.021**	0.11

Blood TG	Total	*y* = 75.5 + 4.97 × (salivary TG)	**<0.001**	0.182
	Case	*y* = 88.67 + 4.8 × (salivary TG)	**0.0018**	0.186
	Control	*y* = 74.7 + 3.79 × (salivary TG)	**0.025**	0.10

Blood HDL-C	Total	*y* = 40 + 2.1 × (Salivary HDL-C)	0.05	0.038
	Case	*y* = 42.37 + 1.12 × (Salivary HDL-C)	0.53	0.008
	Control	*y* = 38.11 + 2.4 × (Salivary HDL-C)	0.09	0.06

Blood LDL-C	Total	*y* = 84 + 2 × (salivary LDL-C)	**0.003**	0.085
	Case	*y* = 79.13 + 2.16 × (salivary LDL-C)	**0.037**	0.088
	Control	*y* = 84.78 + 2.45 × (salivary LDL-C)	**0.02**	0.11

Blood urea	Total	*y* = 11.63 + 0.54 × (salivary urea)	**<0.001**	0.497
	Case	*y* = 13.88 + 0.503 × (salivary urea)	**<0.001**	0.39
	Control	*y* = 14.62 + 0.37 × (salivary urea)	**<0.001**	0.26

Blood creatinine	Total	*y* = 0.43 + 1.5 × (salivary creatinine)	**<0.001**	0.648
	Case	*y* = 0.39 + 1.67 × (salivary creatinine)	**<0.001**	0.39
	Control	*y* = 1.07 + 0.49 × (salivary creatinine)	**<0.001**	0.36

Tc, total cholesterol; TG, triglyceride; HDL-C, high-density lipoprotein cholesterol; LDL-C, low-density lipoprotein cholesterol; *R*^2^ denotes coefficient of determination, and bold indicates the level of significance at *p* ≤ 0.05.

## Data Availability

All the data generated during this study are presented in this paper. The primary raw data will be made available to the interested researchers by the corresponding author of this article if requested.

## Abbreviations

T2DM: Type 2 diabetes mellitus
DM: Diabetes mellitus
WHO: World Health Organisation
IDF: International Diabetes Federation
ROC: Receiver operating characteristic curve
CVD: Cardiovascular disease
CKD: Chronic kidney disease
MMTH: Manmohan memorial teaching hospital
BMI: Body mass index
SBP: Systolic blood pressure
DBP: Diastolic blood pressure
WC: Waist circumference
HC: Hip circumference
TC: Total cholesterol
TG: Triglycerides
HDL-C: High-density lipoprotein cholesterol
LDL-C: Low-density lipoprotein cholesterol
CI: Confidence interval
AGEs: Advanced glycation end products
RAGE: Receptors for advanced glycation end products
PKC: Protein kinase C.
